# The Impact of Leisure Activities on the Mental Health of Older Adults: The Mediating Effect of Social Support and Perceived Stress

**DOI:** 10.1155/2021/6264447

**Published:** 2021-11-08

**Authors:** Chi Zhang, Niu Qing, Sifeng Zhang

**Affiliations:** School of Public Policy and Administration, Xi'an Jiaotong University, No. 28 Xianning West Road, Xi'an 710049, China

## Abstract

As the aging continues, China has become the country with the largest older population. In order to ensure the well-being of older adults in their later years, the whole society is increasingly concerned about the mental health of older adults. In 2019, we conduct a questionnaire survey in Shaanxi Province. Stratified random sampling is used to select three representative cities, and 677 samples are selected from the survey results for research. By using the structural equation model, we aim to reveal the mechanism of leisure activities' influence on mental health of the older adults and verify whether social support and perceived stress play a mediating role. The study finds that the older adults' leisure activities have no significant direct impact on mental health. Social support has a significant mediating effect between leisure activities and mental health of the older adults. Leisure activities indirectly affect the mental health of the older adults through social support, and participation in leisure activities can improve the social support of the older adults, thus improving the mental health level of the older adults. Perceived stress plays a significant mediating role between leisure activities and mental health of the older adults. By participating in leisure activities, the perceived stress of the older adults will be reduced, thus improving their mental health. Social support and perceived stress play a sufficient mediating role in the influence of leisure activities on mental health.

## 1. Introduction

China has become the country with the largest older population in the world. At the end of 2019, China's older population aged 60 and above reached 253.88 million, accounting for 18.1% of the total population, and there will be about 180 million older adults aged 65 and above in China in 2020, accounting for about 13% of the total population [1], which is much higher than the statistical standard of population aging proposed by the United Nations, and China has a deeply aging society. The health problems of older adults have become the focus of attention of the government and society [2]. With the progress of modern medicine and the change of medical model, the concept of health has long been not only physical health but also mental health, both of which are in a perfect state to be called real health [3]. With the increase of age, the physiological and mental functions of older adults gradually decline, which can cause loneliness, anxiety [4]. Negative emotions have a negative impact on the mental health of older adults, and they then affect the quality of life of older adults in their later years; the mental health and negative emotions of older adults have a significant impact on their level of well-being [5].

There are many factors that influence the mental health of older adults, including interpersonal relationships, family factors, and life stress [6]. Currently, a lot of older adults live in the community in their later years. The “one-child” policy has resulted in most families having only one child, and this family structure can leave older adults without care from their children as they age [7]. The current family structure is also leading to a gradual change in the traditional intergenerational relationship; the traditional concept of “serving older adults” is losing its cultural binding force, and the family is lacking in the comforting function of older adults' mental health. Older adults need to participate in leisure activities to enrich their life in their old age [8]. Therefore, the active participation of older adults in leisure activities can effectively meet the spiritual and cultural needs of older adults, promote the harmony of social relationships among older adults, relieve the stress of daily life of older adults, and promote further improvement of the mental health of older adults [9].

With social progress and economic development, older adults' demand for mental health is increasing [10]. Happiness in later life has become the biggest pursuit of older adults [11]. Mental health is the pillar of physical health. If older adults do not have a healthy state of mind and emotion, the body may be reduced or lose its function, leading to diseases [12], and even affecting the life of older adults. Leisure activities have always been an important part of human life and development [13]. In modern society, as older adults have gradually increased their life expectancy, they have higher expectations for the quality of life in their later years, and the importance of maintaining an active lifestyle in their later years has become more prominent [14]. As an important part of the life of older adults, leisure activities are an important factor affecting the health and quality of life of older adults. How to improve the level of participation in leisure activities has also become an important issue to be addressed [15]. Older adults can gain social support, a sense of belonging, fulfillment, and achievement when they participate in leisure activities [16]. Leisure behaviors help older adults to reduce anxiety and cultivate their emotions by communicating with relatives and friends, reducing their perceived stress, and providing them with spiritual comfort [17]; at the same time, adequate leisure activities not only increase older adults' subjective well-being but also improve their positive emotions [18], leading to a more positive and optimistic attitude toward life [19].

## 2. Hypothesis and Framework

With the living standards of older adults continuing to rise, older adults' demand for mental health is increasing [10]. Happiness in old age has become the greatest pursuit of older adults [11]. Mental health is the backbone of physical health. If the older adults do not have a healthy mental and emotional state, physical functions may be reduced or lost, leading to disease [12], and even affecting the quality of life.

About control variables, studies have found that the mental health of older adults is closely related to personal, family, economic, social, and other variables [20]. Loss of a spouse greatly reduces the subjective well-being of older adults, and there is a close relationship between a strong family bond and the emotional well-being of older adults. The degree of disability, sleep duration, chronic disease, and other physiological health variables are also the main factors affecting the mental health of the older adults [21]. Leisure activity can curb depression in older adults and promote longevity [22]. Individual factors such as age, sex, and living in city have no significant influence on the mental health of older adults [23].

Leisure activities are aimed at older adults' leisure, relaxation, pleasure, and development [24]. Studies have shown that reasonable leisure activities contribute to the physical and mental health of older adults and promote their family harmony [25]. Leisure activity can curb depression in older adults and promote longevity [22]. The significance of leisure activities is that it can become an effective way for older adults to pursue self-value and integrate into society [26]. Leisure activities play a good role in venting all kinds of worries and anxieties and promoting mental balance [27].

Social support refers to the help provided by family members, friends, neighbors, and others [28]. In the narrow sense, social support refers to support from outside the family, such as community, relatives, friends, and neighbors [29]. Social support for older adults is also a source of friendship and affection [28]. Participation in social activities, acceptance of social support, and religion may improve the mental status of older adults [30]. Diversified and frequent leisure activities can increase the social relations of older adults and enhance social participation [31, 32]. With the termination of work, the reduction of welfare level, and the narrowing of social circle, the living conditions of older adults are becoming more and more difficult, thus increasing the life pressure of the older adults in their later years [33]. Stress is a long-term existence, through a certain amount of accumulation, with a recurring, intermittent, or persistent mental pattern [34]. Stress can lead to mental illness and damage human health by producing negative consequences such as anxiety, depression, and burnout [35]. The older adults will be more impacted by stress events; the increase of stress events will bring greater pressure to the older adults, and negative emotions will be more intense [36]. Previous studies have shown that perceived stress has a positive predictive effect on depression [37, 38].

We choose escort theory and role optimization reasons as the theoretical basis of this study. Escort model studies how individuals interact with their social network objects and obtain social support and emotional satisfaction at the same time. In order to resist the physical and mental pressure of aging and adapt to the negative emotions brought by the environment, the older adults hope to obtain more intimate feelings and life satisfaction in social communication. According to the social escort model, social support mainly comes from an individual's family, friends, and social network of interpersonal communication, and the social network will change with the change of the individual's living environment [39]. Social network plays an escort role on the individual, especially on the physical and mental health of the older adults, and has a positive role in promoting the mental health of the older adults [40]. Among them, family network is an important source of mental and economic support for the older adults, which can effectively reduce their depression level. Interactions with friends can enhance their sense of self-worth and reduce the risk of psychological discomfort caused by social isolation [41]. Therefore, friend network can address the negative psychological state of the older adults and play an increasingly important protective role in their mental health [42].

At present, domestic researches in China emphasize more on the role of family network, but the discussion on friend network is rare. Generally speaking, in the face of frustration and sense of failure caused by their social status change and physical function decline, the positive problem-oriented coping style can help the older adults to relieve pressure and improve their mental health level. Compared with surfing the Internet, watching movies, and other behaviors, participating in sports, cultural activities, and other recreational activities is more conducive to relieve anxiety and improve mental health of the older adults and they have more time to gather with friends and expand their leisure network.

Role optimization theory suggests that older adults can deepen their roles and enhance their social experiences, and in the process, older adults engage in leisure activities to gain access to richer social resources, such as social networks, which can help them get social support and coping strategies when they encounter stressful events. Role fulfillment also means emotional satisfaction and fullness in health, power, and status [43]. Participating in leisure activities means that older adults engage in social participation, expanding their circle of friends in order to gain greater social support and reduce their stress, which plays a positive role in promoting their mental health.

Through the above theoretical elaboration, the mental health of older adults is influenced by leisure activities, social support, and perceived stress [44]. Therefore, based on the above characteristics, Figure 1 shows the analysis framework of the factors influencing the mental health of older adults established in this article. Leisure activities influence the mental health of older adults, and social support and perceived stress play a mediating role in the process [45, 46].

Combined with the above analysis, the following hypotheses are proposed in this article.

**Hypothesis 1 .**

Leisure activities have a significant impact on the mental health of older adults.

**Hypothesis 2 .**

Social support plays an intermediary role between leisure activities and mental health of the older adults. Participation of the older adults in leisure activities will improve the social support they get, and the mental health level of the older adults will be further improved through the improvement of social support.

**Hypothesis 3 .**

Perceived stress mediates the relationship between leisure activities and mental health in older adults. Older adults who participate in leisure activities have a higher probability of reducing perceived stress and thus improving their mental health.

### 2.1. Data Source

The data of this study come from the field survey of 24 teachers and students in the Social Security Research Center of Xi'an Jiaotong University in 2019. All the authors of this paper participated in this survey.

According to the regional distribution of Shaanxi Province, this field survey adopts stratified random sampling method, selecting Yan'an, Baoji, and Hanzhong as the first layer; randomly selecting 2 counties in each city as the second layer, with a total of 6 counties; then randomly selecting 2 townships from each county as the third layer; and finally randomly selecting 2 communities from each township as the fourth layer, with a total of 24 communities for investigation. The population aged 60 and above accounted for 19.2% in the Shaanxi province, and the population aged 65 and above accounted for 13.32%. The degree of aging in Shaanxi province is similar to the national average. Life expectancy is 77.4 in China and 77.3 in the Shaanxi Province. Shaanxi is a province located in the geographical center of China, and almost all aspects of social economy are at the national average level. Therefore, it is of representative significance to select Shaanxi Province. The survey targets older adults aged 60 and above. Before collecting the data, we orally introduced the background, content, and purpose of the research to the interviewees, and assured them that the data did not involve any personal privacy information, and was only used for research. Only when the interviewees confirm their willingness to participate in this survey will our investigators begin to investigate. All the procedures carried out in the study are in accordance with ethical standards. All questionnaires were completed anonymously after obtaining the oral informed consent of each participant.

A total of 980 questionnaires were distributed, of which 948 were valid. After excluding the samples living in nursing institutions and missing values, we finally selected 677 older adults living in the community.

### 2.2. Variable Selection

The hypothesis testing in this article is based on the theoretical hypothesis model of the factors influencing mental health of older adults constructed in the previous article, selecting mental health of older adults as the (potential) dependent variable, leisure activities of older adults as the (potential) independent variable, and social support and perceived stress as the (potential) mediating variables, and selecting appropriate indicators to measure each variable. Based on previous studies and the theoretical model of this study, the specific variable selection and their descriptive statistics are shown in Table 1.

#### 2.2.1. Dependent Variable: Mental Health

The mental health of the older adults is a complex comprehensive state. We use four variables closely related to mental health in the questionnaire to reflect the mental state of the older adults. These four variables are “1self-evaluation of the current mental state,” “2satisfaction with life,” “3freedom of life” and “4whether the older adults feel lonely” [47].

#### 2.2.2. Independent Variable: Leisure Activities

The variable of leisure activities is reflected by the question, “do you participate in leisure activities in the community,” in the questionnaire. A value of 1 indicates that the older adults participate in the activity, and a value of 0 indicates that the older adults do not participate in the activity. There are seven types of leisure activities, which are interest groups, artistic performances, chess and card activities, knowledge lectures, electronic games, university for the older adults, and sports activities. Finally, the scores of participating in various activities were added up to obtain the leisure activity variable (mean value 1.19, standard deviation 1.210), with a value range of 0–7. The higher the score, the more older adults participate in leisure activities provided by the community.

#### 2.2.3. Intermediary Variables: Social Support and Perceived Pressure

Social support mainly refers to the support from friends that older adults receive. Through “Are you in a harmonious relationship with friends in your neighborhood (older adults) (mean: 4.32, standard deviation: 0.785),” “Do you and friends in your neighborhood (older adults) often help each other (mean: 4.12, standard deviation: 0.921),” “Do you and your friends often chat together (mean: 4.28, standard deviation: 0.994)” three observation variables are measured, and each observation variable is measured by the Likert scale. The table is scored, and the value is 1–5.

Perceived stress refers to various life stresses such as physical health, economic problems, and care problems. A higher score of perceived stress indicated a lower stress level. Through “If you cannot take care of yourself, do you worry about being unattended (mean: 3.36, standard deviation: 1.496)?,” “whether you are worried about not having money in the future (mean: 3.11, standard deviation: 1.379)?,” “the main illness that currently bothers you (mean: 3.24, standard deviation: 0.569),” “how is your physical condition (mean: 3.47, standard deviation: 1.084)>” four observation variables are measured. Among them, “If you cannot take care of yourself, are you worried about being left unattended?,” “whether you are worried that you will have no money in the future?,” “what is your physical condition?,” “The main illness that currently bothers you” refers to the five categories of diseases that the older adults may suffer from at present, including chronic diseases, mental diseases, disabilities, diseases requiring hospitalization, and senile diseases. For multiple choice questions, one point is awarded for each choice selected, and the total scores are summed up, with a total score ranging from 0 to 5.

### 2.3. Sample Description

Table 2 shows the statistical characteristics for the sample of this survey. Among the surveyed older adults, the youngest is 60 years old and the oldest is 92 years old, with an average age of 70.40 years old; the ratio of men to women is about 0.63 : 1, with more female older adults than male older adults; in terms of education level, 43.1% of older adults have elementary school education or less, and only about 8% have college education or above, so the overall education level of the surveyed older adults is low; in terms of household registration, the ratio of urban and rural households is 1.35 : 1; in terms of living style, the ratio between older adults living alone and those not living alone is 0.23 : 1; in terms of self-care ability, the mean value of ADL was 0.05, meaning that the majority of older adults are not physically impaired; in terms of marriage type, the largest number of older adults are married, accounting for 71.6%, followed by widowed, accounting for 25.4%, which is one-fourth of the total number of older adults surveyed; in terms of pre-retirement employment, farmers and employees of enterprises and institutions accounted for the largest proportion, with 39.9% and 39.7%, respectively.

### 2.4. Analysis Method

SPSS20.0 is used for data preprocessing and simple descriptive statistics, and AMOS24.0 is used for mediating effect analysis using structural equation model.

Structural equation models include: (1) Measurement model: reflecting the relationship between latent variables and observed variables. The so-called observed variables are the data obtained by measurement tools such as scales or questionnaires, while the latent variables are the characteristics or abstract concepts formed among the observed variables, which cannot be directly measured and need to be reflected by the measured data of the observed variables. (2) Structural model: it reflects the causal relationship between latent variables. The criteria for a good model: GFI > 0.9, AGFI > 0.9, NFI > 0.9, IFI > 0.9, TLI > 0.9, PGFI > 0.5, PNFI > 0.5, CMIN/DF < 5.052.

## 3. Results

### 3.1. Reliability and Validity Tests

With the help of SPSS20.0 and AMOS24.0 software, standardized factor load, internal consistency reliability coefficient (Cronbach's Alpha value), combined reliability (CR), and mean variance extraction (AVE) were used to measure the convergence validity of each potential variable in the model, and the test results are shown in Table 3. As shown in Table 3, the limit of standardized factor load of each observation variable was between 0.508 and 0.918, all of which were greater than 0.5, indicating that the basic adaptation index of the scale was ideal. The internal consistency reliability coefficients (Cronbach's Alpha value) of each potential variable were 0.846, 0.601, and 0.791, respectively. The combined reliability (CR) of the potential variables were 0.854, 0.639, and 0.796, respectively. The average variance extraction (AVE) of each potential variable was 0.663, 0.308, and 0.498, respectively, which indicated that each potential variable of the model had good convergence validity and good reliability [48].

Mean variance extraction (AVE) was used to test the discriminant validity of the model. If the square root of the AVE value of each potential variable was greater than the absolute value of the correlation coefficient between it and other potential variables, the variables were considered to have good discriminant validity [49]. The results of discriminant validity analysis are shown in Table 4. Table 4 shows that the square root of AVE value of each potential variable is higher than the absolute value of its correlation coefficient with other potential variables, indicating that the model has good discriminative validity among potential variables.

### 3.2. Model Fit Test

In this article, the degree of fit of the constructed structural equation model was tested using 11 fit indices in terms of absolute fitness index, value-added fitness index, and parsimony fitness index, and the test results are shown in Table 5. In Table 5, the GFI value was 0.948, which was greater than 0.9; the AGFI value was 0.919, which was greater than 0.9; the NFI, IFI, TLI values range from 0.907 to 0.930, which were all greater than 0.9; the PGFI value was 0.608, which was greater than 0.5; the PNFI value was 0.691, which was greater than 0.5; and the cardinality freedom ratio CMIN/DF was 4.495, which was less than 5. The comprehensive data above showed that all the fitting indicators meet the acceptable criteria, indicating that the constructed structural equation model had a high overall fit with the data, the model fitness was good, the model did not need to be revised, and the initial theoretical model was used as the final accepted model.

### 3.3. Path Analysis and Hypothesis Testing

Structural equation analysis of mental health influencing factors of older adults was conducted using AMOS24.0 software, and Figure 2 shows the schematic diagram of the structural equation model of mental health influencing factors of older adults. To investigate the indirect effects of mediating variables on the dependent variable, this article obtained percentile bootstrapping and bias-corrected percentile bootstrapping by using the Bootstrap procedure with 5000 replicate samples at 95% confidence intervals and estimation by the great likelihood method. If percentile bootstrapping and bias-corrected percentile bootstrapping contains 0, the mediation effect of this result was not significant:

1. Table 6 shows the results of the model path coefficient test, and Table 7 shows the results of the model mediation effect test. As can be seen from Tables 6 and 7, the nonstandardized path coefficient of the direct effect of leisure activities on the mental health of older adults was 0.024, with a *p* value of 0.394, which was greater than 0.05, and H1 failed the test, which indicates that leisure activities could not directly affect the mental health of older adults, and social support and perceived stress played a complete mediating effect between leisure activities and the mental health of older adults.
2. As shown in Table 6, the nonstandardized path coefficient between leisure activities and social support was 0.146, and the *p* value was less than 0.001; the nonstandardized path coefficient between social support and older adult's mental health was 0.431, and the *p* value was less than 0.001. Meanwhile, as shown in Table 7, the mediating effect of social support between leisure activities and older adults' mental health was significant (Bias-corrected 95% CI: Lower = 0.034, Upper = 0.100; Percentile 95% CI: Lower = 0.033, Upper = 0.098). The above results suggested that leisure activities indirectly affect the mental health of older adults through social support, and Hypothesis 2 was verified.
3. As shown in Table 6, the nonstandardized path coefficient between leisure activities and perceived stress was 0.093, with *p* value less than 0.05; the nonstandardized path coefficient between perceived stress and mental health of older adults was 0.435, with *p* value less than 0.001. Meanwhile, as shown in Table 7, the mediating effect of perceived stress between leisure activities and mental health of older adults was significant (Bias-corrected 95% CI: Lower = 0.003, Upper = 0.084; Percentile 95% CI: Lower = 0.001, Upper = 0.082). The above results suggested that leisure activities indirectly affect the mental health of older adults through perceived stress, and Hypothesis 3 was tested.

## 4. Discussion

### 4.1. Leisure Activities Have Significant Effects on Social Support and Perceived Stress of Older Adults

Leisure activities are an important part of the daily life of older adults and an important factor in maintaining the subjective well-being and life satisfaction of retired older adults [15, 50]. This study shows that leisure activities have significant effects on social support, perceived stress. and mental health of older adults, and the importance of leisure activities for older adults should be strengthened. In the context of China's aging population, leisure activities are an important way for older adults to participate in social activities and have a positive effect on their mental health and social well-being [51].

The use of leisure activities can expand older adults' social support, reduce perceived stress, and positively contribute to their mental health [52, 53]. The role optimization theory suggests that a variety of roles will provide older adults with more fulfilling roles and enhance their social experiences, in which they will gain richer access to important resources such as social networks and social support during stressful events [54], as confirmed by the results of this study.

Role optimization theory is put to good use in this paper, which found that older adults who participate in leisure activities have more opportunities to interact with their friends, and these opportunities expand and optimize their social networks and daily communication, promoting the continuation of friendships and thus alleviating depression levels. The older adults who participate in leisure activities have more common topics among themselves, thus expanding their network of friends. Participation in leisure activities enables the older adults to have a more fulfilling daily life, improve their sense of self-efficacy and self-worth, make them feel more fulfilling and meaningful life, and reduce their depressive symptoms.

After retirement from society to family, older adults are missing social participation roles and social contact is reduced, which makes them prone to loneliness, low self-esteem, frustration, and other negative emotions [55]. Participating in leisure activities can provide opportunities for older adults to interact with other older adults, thus expanding their friend networks, making up for their missing social participation due to retirement from work, and satisfying their sense of value. When older adults encounter financial difficulties, they are more likely to be assisted by people they know through leisure activities, because leisure activities enable them to share common interests and form deep friendship, even if their older peers do not have the money to help, their language and behavior will play a comforting role to lighten older adults' mood, and greatly reduce the older adults' depression levels.

### 4.2. Social Support and Perceived Stress Play a Mediating Role between Leisure Activities and Older Adults' Mental Health

The results of this article show that social support, perceived stress play a fully mediating role between leisure activities and older adults' mental health, and that leisure activities can reduce the risk of depression and maintain mental health by expanding social support and reducing perceived stress. The results suggest that, on the one hand, using leisure activities makes older adults more likely to have a stronger network of friends and receive more social support, thus reducing the risk of depression and maintaining their mental health, which is consistent with the social escort theory and the main effect model of social support [39, 56–58]. On the other hand, the use of leisure activities can improve the physical health of older adults, enhance their ability to resist various risks, reduce their perceived stress, and thus reduce their depressive symptoms and improve their mental health [59].

Since social support and perceived stress play a mediating role between leisure activities and older adults' mental health, the effect of leisure activities on older adults' mental health must be realized through social support and perceived stress. The increase of social support and the decrease of perceived stress will reduce the probability of poor mental health in the older adults. On the one hand, communities can organize more leisure and recreational activities to increase social interaction opportunities for older adults, and further expand the network of friends and improve the quality of social networks. On the other hand, communities should carry out leisure and recreational activities that are beneficial to the physical health of older adults and enhance their physical health through participation in leisure and recreational activities, thus reducing their perceived stress.

On this basis, communities should change the previous and “service-centered” development mindset to a “demand-centered” approach. “In addition to carrying out leisure activities, we should conduct demand surveys and assessments, and strive to supply leisure activities from the perspective of the actual needs of older adults, so as to increase the frequency of leisure activities for older adults and improve their mental health. By strengthening the paths of “leisure activities-social support” and “leisure activities-perceived stress,” the ultimate goal is “leisure activities-social support-mental health.” The path of “leisure activity-perceived stress-mental health” can fully realize the positive effect of leisure activities on the mental health of older adults.

## 5. Conclusions

This article builds an analytical framework of leisure activities, social support, perceived stress, and mental health of older adults, and it empirically analyzes the effects of leisure activities on the mental health of older adults by applying structural equation modeling using data from a field study in Shaanxi Province in 2019. It is found that leisure activities have significant effects on social support, perceived stress, and mental well-being of older adults. The article further explores the mediating role of social support and perceived stress between leisure activities and older adults' mental health, and the results show that social support and perceived stress fully mediate the relationship between leisure activities and older adults' mental health, and that leisure activities reduce the risk of depression and maintain older adults' mental health by expanding social support and reducing perceived stress.

Older adults in this study mainly live in the community, and there is a lack of research on older adults living in nursing homes. In the future, the impact of leisure activities on the mental health of older adults living in nursing homes can be studied, because there are great differences between older adults living in nursing homes and those living in the community. Due to the existence of the urban-rural dichotomy in China, the leisure activities and mental states of the urban and rural older adults also differ greatly, which is also a direction worth studying in the future. Finally, the content of leisure activities of older adults has been greatly transformed in the context of the COVID-19, and how to reconsider the leisure activities of older adults in the context of the COVID-19 is a topic worth considering. Potential limitations of this paper are that the data selected are cross-sectional data, and we currently do not have a good way to demonstrate the direction of the effects of the variables selected in the paper. Similarly, although researchers do sometimes test mediation in cross-sectional data, methodologists often view this as not a valid approach. Demonstrating the direction of the effects of the variables selected in the paper is a worthy study in the future.

## Figures and Tables

**Figure 1:** Framework for analyzing factors influencing mental health of older adults.

**Figure 2:** Structural equation model of mental health of older adults.

**Table 1:** Descriptive statistics of variables.

Latent variable	Question	Number	Definition	Mean	Standard deviation
Leisure activities	To participate in leisure activities	A1	0–7	1.19	1.210
Social support	Do you have a good relationship with your neighbors and friends?	B1	1 = very discordant; 2 = disharmony; 3 = in general; 4 = more harmonious; 5 = very harmonious	4.32	0.785
	Do you often help each other with your neighbors and friends?	B2	1 = never; 2 = mostly not; 3 = generally; 4 = often; 5 = always	4.12	0.921
	Do you often have activities and chat with neighbors and friends?	B3	1 = never; 2 = mostly not; 3 = generally; 4 = often; 5 = always	4.28	0.994

Perceived stress	Are you worried about being left unattended?	C1	1 = very worried; 2 = quite worried; 3 = fairly worried; 4 = not worried; 5 = not worried at all	3.36	1.496
	Worrying about having no money for the future	C2	1 = very worried; 2 = quite worried; 3 = fairly worried; 4 = not worried; 5 = not worried at all	3.11	1.379
	Main illness	C3	0–5	3.24	0.569
	Physical condition	C4	1 = very poor; 2 = poor; 3 = fair; 4 = better; 5 = very good	3.47	1.084

Mental health	Satisfaction with life condition	D1	1 = very dissatisfied; 2 = dissatisfied; 3 = fair; 4 = more satisfied; 5 = very satisfied	4.00	0.904
	Freedom of life	D2	1 = very unfree; 2 = not free; 3 = fair; 4 = more free; 5 = very free	4.34	0.789
	Whether the older adults feel lonely	D3	1 = always; 2 = often; 3 = sometimes; 4 = rarely; 5 = never	4.00	0.984
	Self-evaluation of the current mental state	D4	1 = very poor; 2 = poor; 3 = fair; 4 = better; 5 = very good	4.19	0.931

**Table 2:** Statistical characteristics of the samples.

Variables	Classification	Number	Frequency (%)
Age	60 years old and above	Mean value.70.41; standard deviation.7.08	

Gender	Male	261	38.6
	Female	416	61.4

Education	Elementary school	292	43.1
	Junior high school	193	28.5
	High school/junior high school	137	20.2
	College	38	5.6
	Bachelor's degree or above	17	2.5

Marriage	Unmarried	10	1.46
	Married	489	71.60
	Divorced	10	1.46
	Widowed	174	25.48

Household registration	Urban	389	57.5
	Rural	288	42.5

Whether living alone	No	551	81.4
	Yes	126	18.6

Pre-retirement work	Civil servants	43	6.4
	Employees of enterprise units	269	39.7
	Individual operators	20	3.0
	Farmers	270	39.9
	Migrant workers	26	3.8
	Others	49	7.2

Activities of daily living (ADL)	0∼6	Mean value.0.05; standard deviation.0.43	

**Table 3:** Convergent validity test results.

Latent variable	Number	Parameter significance estimation				Factor load	Composite reliability	Average variance extraction	Cronbach's alpha
		Unstd.	SE	*t*-value	*p*	Std.	CR	AVE	
Leisure activities	A1	0.880				0.727	—	—	—

Social support	B1	1.000				0.757	0.854	0.663	0.846
	B2	1.422	0.070	20.384	^*∗∗∗*^	0.918			
	B3	1.264	0.065	19.541	^*∗∗∗*^	0.756			

Perceived stress	C4	1.000				0.598	0.639	0.308	0.601
	C3	0.510	0.058	8.728	^*∗∗∗*^	0.581			
	C2	1.121	0.133	8.458	^*∗∗∗*^	0.528			
	C1	1.171	0.141	8.306	^*∗∗∗*^	0.508			

Mental health	D1	1.000				0.598	0.796	0.498	0.791
	D2	0.933	0.073	12.714	^*∗∗∗*^	0.639			
	D3	1.318	0.096	13.764	^*∗∗∗*^	0.724			
	D4	1.443	0.101	14.337	^*∗∗∗*^	0.838			

*Note*. The symbol ^*∗∗∗*^ means significant at the 0.1% level, ^*∗∗*^ means significant at the 1% level, and ^*∗*^ means significant at the 5% level.

**Table 4:** Differential validity test results.

	Social support	Leisure activities	Mental health	Perceived stress
Social support	**0.814**			
Leisure activities	0.225	**0.727**		
Mental health	0.553	0.212	**0.706**	
Perceived stress	0.204	0.109	0.603	**0.555**

*Note*. The value on the diagonal represents the square root of AVE, and the value below the diagonal is the correlation coefficient among the potential variables.

**Table 5:** Model fit test results.

Fit index classification		Model fit value test results	Standard	Fit result
Absolute fit index	GFI	0.948	>0.9	Perfect
	AGFI	0.919	>0.9	Perfect

Value-added fitness index	NFI	0.912	>0.9	Perfect
	IFI	0.930	>0.9	Perfect
	TLI	0.907	>0.9	Perfect

Simplicity fit index	PGFI	0.608	>0.5	Perfect
	PNFI	0.691	>0.5	Perfect
	CMIN/DF	4.495	<5.0	Perfect

**Table 6:** Model path coefficient test.

Path	Nonstandardized coefficient	SE	CR	*p*	Results
Leisure activities ⟶ perceived stress	0.093	0.043	2.139	^*∗*^	Significant
Leisure activities ⟶ social support	0.146	0.035	4.170	^*∗∗∗*^	Significant
Perceived stress ⟶ mental health	0.435	0.053	8.224	^*∗∗∗*^	Significant
Social support ⟶ mental health	0.431	0.044	9.707	^*∗∗∗*^	Significant
Leisure activities ⟶ mental health	0.024	0.029	0.852	0.394	Not significant

*Note*. The symbol ^*∗∗∗*^ means significant at the 0.1% level, ^*∗∗*^ means significant at the 1% level, and ^*∗*^ means significant at the 5% level.

**Table 7:** Tests of mediating effects on mental health of older adults.

	Point estimation	Product of coefficients		Bootstrapping			
				Bias-corrected 95% CI		Percentile 95% CI	
		SE	*Z*	Lower	Upper	Lower	Upper
*Indirect effects*							
Leisure activities ⟶ social support ⟶ mental health	0.063	0.016	3.938	0.034	0.100	0.033	0.098
Leisure activities ⟶perceived stress ⟶ mental health	0.040	0.021	1.905	0.003	0.084	0.001	0.082
Total indirect effect	0.103	0.030	3.433	0.047	0.168	0.044	0.165

*Direct effect*							
Leisure activities ⟶ mental health	0.024	0.029	0.828	−0.033	0.082	−0.032	0.084
*Total effect*							
Leisure activities⟶ mental health	0.128	0.034	3.765	0.064	0.197	0.063	0.197

*Note*. 5000 bootstrap samples.

## Data Availability

The data used in this study can be obtained from the corresponding author upon reasonable request.
